The article "Hopeless tooth and less posterior occlusion is related to a greater risk of low handgrip strength: A population-based cross-sectional study" was published in 2021. Journal: PLoS One.

# Hopeless tooth and less posterior occlusion is related to a greater risk of low handgrip strength: A population-based cross-sectional study

**DOI:** 10.1371/journal.pone.0260927

**Published:** 2021-12-23

**Authors:** Sul-Hee Kim, Xianhua Che, Hee-Jung Park, Tae-Il Kim

**Affiliations:** 1 Dental Research Institute, Seoul National University School of Dentistry, Seoul, Korea; 2 Department of Health Policy Research, Daejeon Public Health Policy Institute, Daejeon, Korea; 3 Department of Dental Hygiene, Kangwon National University, Samcheok, Korea; 4 Department of Periodontology, Seoul National University School of Dentistry, Seoul, Korea; School of Dentistry, International Medical University, MALAYSIA

## Abstract

The effect of severely compromised teeth on masticatory function has not been properly evaluated in previous studies, as they were often considered equivalent to the healthy tooth or excluded as if absent in the dentition. Hopeless teeth, which refer to non-salvageable teeth that require extraction, can interfere with masticatory function. As posterior occlusion is directly related to the masticatory function, we evaluated pairs opposing posterior teeth (POPs) that reflect the arrangement as well as the number of remaining posterior teeth. This study investigated the relationship of a hopeless tooth to handgrip strength according to POPs in the elderly. This cross-sectional study used data from the Korea National Health and Nutrition Examination Survey (KNHANES). Among the data of 23,466 participants from 2015 to 2018, participants aged 60 years or older (n = 4,729) were included. In males with POPs scores of 0–7, considered poor posterior occlusion, the association with low handgrip strength persisted in the multivariate logistic regression model adjusted for all confounding variables. The odds ratio (OR) in the absence of hopeless teeth (OR = 1.91, 95% CI: 1.02–3.59) increased in the presence of a hopeless tooth (OR = 2.78, 95% CI: 1.42–5.47). Even with POPs scores of 8–11, considered good posterior occlusion, the association was significantly high in the presence of a hopeless tooth (OR = 2.82, 95% CI: 1.06–7.52). In females, the association disappeared in adjusted models. The fewer pairs of natural posterior teeth with occlusion, the greater the risk of low handgrip strength. Dentition containing hopeless teeth increases the risk of low handgrip strength, even in dentition with sufficient posterior occlusion. Preserving the posterior teeth in a healthy condition through personal oral hygiene and regular dental management is essential for maintaining components of physical function such as handgrip strength.

## Introduction

The elderly population is increasing in many countries, and by 2050, the number of people aged 60 or older is expected to account for more than 20 percent of the world’s population [1]. Since the health problems of the elderly population are related to quality of life and can increase socio-economic burden, it is important to evaluate modifiable risks and implement evidence-based efforts to manage and prevent the decline of capacity [2,3].

The article "Hopeless tooth and less posterior occlusion is related to a greater risk of low handgrip strength: A population-based cross-sectional study" was published in 2021. Journal: PLoS One.

Recently, there has been a growing interest in the concept of frailty. This is an age-related syndrome that increases sensitivity to stressors physiologically, functionally, and mentally, causing adverse health outcomes [4,5]. Sarcopenia is considered a precursor to or physical aspect of frailty [6]. Handgrip strength is one of the objective indicators used to screen for frailty and sarcopenia [2,7], and has also been added to the key diagnostic characteristics for sarcopenia [7]. Previous studies have suggested that low handgrip strength can be a clinical marker for weakened physical function and poor mental health, and can predict all-cause mortality [8].

Studies have reported the association between handgrip strength and various factors related to oral conditions such as periodontitis, number of teeth, chewing ability, occlusal force, oral hygiene behavior, and prosthetic type [9–15]. Handgrip strength has been found to be mainly related to mastication. The number of residual teeth, occluding pairs (OPs) and functional tooth units (FTUs) have been used to evaluate masticatory function [16]. OPs for the arrangement of residual teeth are calculated as the number of occlusion of upper and lower teeth [17]. It is generally evaluated to be a more descriptive index for assessing masticatory functioning compared to the number of residual teeth [18]. The FTUs, a concept developed from OPs, show the condition of the teeth and only functional posterior teeth are included in calculation of the number of FTUs [19–23]. Severely compromised teeth that can be considered non-functional were evaluated inconsistently according to the applied concepts in previous studies. When evaluating masticatory function by the number of residual teeth or the OPs, severely compromised teeth were considered equivalent to healthy teeth, and when evaluating masticatory function by the FTUs, severely compromised teeth were excluded as if they did not exist in the dentition.

Periodontal disease or dental caries has a considerably high prevalence, so it is necessary to evaluate the dentition compromised by these diseases from a clinical point of view. In particular, when the teeth that are severely compromised by these diseases are retained in the dentition, discomfort induced by pain or mobility from these teeth can hinder other functional teeth from chewing efficiently. Moreover, the effects on the whole body as well as the masticatory performance may be different compared to when the dentition is composed of only teeth of healthy status.

The article "Hopeless tooth and less posterior occlusion is related to a greater risk of low handgrip strength: A population-based cross-sectional study" was published in 2021. Journal: PLoS One.

However, the effect of severely compromised teeth on mastication remains poorly understood. Therefore, this study focused on teeth severely compromised by periodontitis and dental caries that will require extraction (hopeless teeth) and the objective of this study is to evaluate the effect of hopeless teeth on handgrip strength according to posterior occlusion in the elderly from nationally representative data.

## Materials and methods

### Study population

This study used 2015–2018 data from the Korea National Health and Nutrition Examination Survey (KNHANES). KNHANES is a national survey on health status, health-related awareness and behavior, and food and nutrition intake. Data corresponding to 23,466 participants were merged, and 12,805 participants with missing data were eliminated. In the final sample, 4,729 participants (2,217 males and 2,512 females) aged 60 years or older were included. Since KNHANES have been conducted with IRB exemption under the Bioethics Act since 2015, the institutional review board (IRB) approval was not required [10]. All participants agreed to written informed consent in advance of the examination, and original data accessible to the public was used in this study.

### Posterior occlusion and hopeless teeth

The posterior occlusion was assessed in pairs of opposing posterior teeth (POPs) and scored based on the calculation method of the FTUs. The difference was that for calculation of FTUs, the non-functional teeth were excluded while the hopeless teeth were not excluded in this study. The POPs were scored with the natural posterior teeth excluding missing teeth and third molar teeth. Artificial teeth such as implants, bridges, pontics, and dentures were not included. The POPs score was calculated, assigning 1 point to each pair of opposing premolars and 2 points to each pair of opposing molars. If all natural teeth remained in the posterior area, the score was 6 points on one side and 12 points on both sides. The score had a range of 0–12 points depending on the number and arrangement of remaining posterior teeth [21].

A previous study reported that all foods could be chewed with at least 7.6 natural FTUs [19]. Based on this, participants in the present study were classified into three groups for analysis according to the number of POPs as follows: Poor (0–7 POPs), Good (8–11 POPs) and Complete (12 POPs) [21].

Dental treatment needs are documented in the KNHANES data. The severity of dental need is recorded according to the tooth with the highest score of treatment needs. The codes 1~5 are used where a tooth shows/requires restorative, crown restoration, pulpal and restorative treatment. Codes 6 and 7 are for dental treatment needs that indicate a tooth in a severely compromised state due to dental caries and periodontal disease, respectively. Code 6 should be used to record a condition at an irrecoverable level of severe caries after restorative treatment. In addition, Code 7 is considered as periodontal disease with severe mobility that is judged to be incurable and requires extraction.

The article "Hopeless tooth and less posterior occlusion is related to a greater risk of low handgrip strength: A population-based cross-sectional study" was published in 2021. Journal: PLoS One.

### Handgrip strength

Handgrip strength was measured using a digital dynamometer (Takei Digital Grip Strength Dynamometer Model T.K.K.540, TAKEI, Japan). Measurements were made three times, first with the dominant hand, then alternately with both hands. If there was a functional limitation that made it difficult to measure the force of the handle, as identified through an examination and interview, the case was excluded. The unit of measurement is kilograms (kg). The maximum handgrip strength of the dominant hand was used in the analysis. According to the Asian Working Group for Sarcopenia, low handgrip strength was defined as less than 26 kg in men and less than 18 kg in women [24].

### Confounding variables

The confounding variables used in this study were age, household income, education level, fasting blood glucose, body mass index (BMI), high-sensitivity C-reactive protein (hs-CRP), hypertension, sedentary time, muscular exercise, drinking, smoking, and denture status.

Age was classified into three groups: 1) 60–69, 2) 70–79, 3) 80 years old or older. Household income was classified into four groups: 1) low, 2) low-middle, 3) middle-high, 4) high. Education level was classified into four groups: 1) elementary school, 2) middle school, 3) high school, 4) university or higher. Fasting glucose levels were classified into three groups: 1) normal (<100 mg/dL), 2) pre-diabetes (100–126 mg/dL), and diabetes (≥126 mg/dL). BMI was classified into three groups: 1) <23 kg/m^2^, 2) 23–25 kg/m^2^, 3) ≥25 kg/m^2^. Hs-CRP levels were dichotomized: 1) normal (<1.0 mg/L), 2) high (≥1.0 mg/L) [25]. Blood pressure was classified into three groups: 1) normal (systolic blood pressure <120 mmHg, diastolic blood pressure <80 mmHg, 2) pre-hypertension (systolic blood pressure 120–140 mmHg, diastolic blood pressure 80–90 mmHg), 3) hypertension (systolic blood pressure ≥140 mmHg, diastolic blood pressure ≥90 mmHg). Sedentary time (hours per day) was classified into four groups as follows: 1) <4.7, 2) 4.7–7.4, 3) 7.4–9.9, 4) ≥9.9 [14]. Muscular exercise (days per week) was classified into three groups according to frequency: 1) 0–2, 2) 3–4, 3) ≥5. Drinking (glasses at a sitting) was classified into four groups according to intake quantity at a sitting: 1) non-drinking, 2) 1–4, 3) 5–9, 4) ≥10. Smoking was classified into three groups: 1) non-smoker, 2) former smoker, and 3) current smoker. Denture status was dichotomized according to the use of removable dentures.

The article "Hopeless tooth and less posterior occlusion is related to a greater risk of low handgrip strength: A population-based cross-sectional study" was published in 2021. Journal: PLoS One.

### Statistical analysis

The KNHANES is a survey with a complicated design, including stratification and multistage probability sampling. The weighting of the survey samples were calculated by taking into account the sampling rate, response rate, and age/sex proportions of the reference population (2005 Korean National Census Registry). According to statistical guidelines from the KDCA (Korean Disease Control and Prevention Agency), survey sample weights were used in all analyses to produce a new integrated dataset from the 4-year data that were representative of the noninstitutionalized civilian population. All stratified analyses by gender were conducted to compare handgrip strength. The distributional differences in handgrip strength by gender according to the general characteristics of the study population were used in a chi-squared test. The number of teeth and POPs by age group (60–69, 70–79 and ≥80 years old) are presented as mean ± standard error in one-way analysis of variance (ANOVA). Low handgrip strength in accordance with POPs with or without hopeless teeth was also compared. A multivariate logistic regression analysis was used to evaluate the odds ratios with 95% confidence intervals (CI) of low handgrip strength according to POPs and hopeless teeth. Multivariate regression Model 1 was adjusted for age, household income, and education. Model 2 was adjusted for the confounding variables in Model 1 plus fasting blood glucose, BMI, hs-CRP, blood pressure, sedentary time, muscular exercise, drinking, smoking, and denture status.

All of the tests were 2-sided, and *P*-values <0.05 were considered to indicate statistical significance. Analyses were performed using a statistical software program (STATA 15, StataCorp LP., Texas, USA).

## Results

Table 1 presents the general characteristics of study participants according to their handgrip strength. Participants with low handgrip strength showed a higher distribution compared to participants with normal handgrip strength in older age, lower education level, hypertension, longer sedentary time, lower frequency of muscular exercise, less drinking, and denture use in both males and females. In females, the distribution of low handgrip strength was low when the household income was high, and similar distribution was observed in other income-related subgroups. The distribution of high levels of hs-CRP was higher with low handgrip strength than normal handgrip strength, and the distribution was highest for non-smokers in the normal and low handgrip strength groups, in females. Regarding BMI, males with low handgrip strength showed a higher distribution in <23 kg/m^2^, and females with low handgrip strength showed a higher distribution in <23 kg/m^2^ and ≥25 kg/m^2^.

The article "Hopeless tooth and less posterior occlusion is related to a greater risk of low handgrip strength: A population-based cross-sectional study" was published in 2021. Journal: PLoS One.

**Table 1:** Numbers (%) of subjects with low and normal handgrip according to general characteristics.

Variables	Male				Female			
	N	Low handgrip strength	Normal	*P*-value	N	Low handgrip strength	Normal	*P*-value
**Age (years old)**								
60–69	1,220	56 (19.4)	1,164 (60.2)	<0.001	1,348	195 (29.6)	1,153 (63.4)	<0.001
70–79	802	115 (45.2)	687 (34.1)		937	316 (49.8)	621 (32.2)	
≥80	195	84 (35.4)	111 (5.7)		227	144 (20.6)	83 (4.4)	
**Household income**								
Low	517	74 (28.7)	443 (22.3)	0.085	585	175 (26.7)	410 (22.5)	0.007
Middle-low	570	75 (27.3)	495 (24.0)		636	181 (27.6)	455 (24.7)	
Middle-high	547	53 (21.9)	494 (25.2)		652	156 (25.6)	496 (24.9)	
High	583	53 (22.1)	530 (28.5)		639	143 (20.1)	496 (27.9)	
**Education level**								
Elementary school	772	145 (56.3)	627 (32.1)	<0.001	1,548	503 (76.3)	1,045 (55.7)	<0.001
Middle school	408	35 (12.6)	373 (18.0)		410	81 (11.7)	329 (17.5)	
High school	593	50 (19.6)	543 (27.7)		376	43 (7.1)	333 (18.3)	
College or higher	444	25 (11.5)	419 (22.2)		178	28 (4.9)	150 (8.5)	
**Fasting blood glucose**								
Normal	925	116 (47.1)	809 (41.5)	0.062	1,285	316 (46.9)	969 (51.6)	0.154
Pre-diabetes	893	89 (32.6)	804 (41.8)		866	231 (37.1)	635 (34.9)	
Diabetes	399	50 (20.3)	349 (16.7)		345	103 (16.0)	242 (13.5)	
**Body mass index (kg/m** ^**2**^ **)**								
<23	792	135 (52.7)	657 (33.4)	<0.001	842	248 (38.6)	594 (32.2)	0.019
23–25	638	72 (29.6)	566 (29.0)		630	149 (20.9)	481 (25.7)	
≥25	787	48 (17.7)	739 (37.6)		1,040	258 (40.5)	782 (42.1)	
**High-sensitivity C-reactive protein**								
Normal	1,420	148 (60.3)	1,272 (65.1)	0.202	1,716	395 (62.6)	1,321 (70.3)	0.002
High	797	107 (39.7)	690 (34.9)		796	260 (37.4)	536 (29.7)	
**Blood pressure**								
Normal	434	54 (21.4)	380 (19.7)	0.009	511	91 (14.5)	420 (23.2)	<0.001
Pre-hypertension	512	39 (14.3)	473 (24.4)		514	129 (19.6)	385 (21.7)	
Hypertension	1,271	162 (64.3)	1,109 (55.9)		1,487	435 (65.9)	1,052 (55.1)	
**Sedentary time (hours/day)**								
<4.7	443	30 (11.7)	413 (21.0)	0.001	419	79 (11.5)	340 (18.9)	<0.001
4.7–7.4	679	70 (25.9)	609 (31.3)		762	179 (27.4)	583 (30.2)	
7.4–9.9	375	53 (22.3)	322 (15.8)		425	114 (19.0)	311 (17.4)	
≥9.9	720	102 (40.1)	618 (31.9)		906	283 (42.1)	623 (33.5)	
**Muscular exercise (days/week)**								
≤2	1,654	213 (85.0)	1,438 (72.8)	<0.001	2,289	623 (94.8)	1,666 (90.3)	0.014
3–4	181	13 (5.0)	168 (8.7)		100	15 (2.0)	85 (4.3)	
≥5	382	26 (10.0)	356 (18.5)		123	17 (3.2)	106 (5.4)	
**Drinking (glasses at a sitting)**								
None	606	113 (44.5)	493 (24.6)	<0.001	1,414	435 (68.2)	979 (51.9)	<0.001
1–4	960	108 (40.5)	852 (42.9)		1,032	214 (31.0)	818 (44.5)	
5–9	541	30 (11.7)	511 (27.2)		58	5 (0.7)	53 (3.1)	
≥10	110	4 (3.3)	106 (5.3)		8	1 (0.1)	7 (0.5)	
**Smoking**								
Non-smoker	449	61 (22.0)	388 (19.1)	0.498	2,375	618 (94.4)	1,757 (94.7)	<0.001
Former smoker	1,316	143 (59.4)	1,173 (59.7)		79	22 (3.3)	57 (3.1)	
Current smoker	452	51 (18.6)	401 (21.2)		58	15 (2.3)	43 (2.2)	
**Denture status**								
No	1,748	166 (65.5)	1,582 (80.9)	<0.001	2,067	476 (72.5)	1,591 (85.4)	<0.001
Yes	469	89 (34.5)	380 (19.1)		445	179 (27.5)	266 (15.6)	

Values are presented as number (weighted percent).

The article "Hopeless tooth and less posterior occlusion is related to a greater risk of low handgrip strength: A population-based cross-sectional study" was published in 2021. Journal: PLoS One.

*P*-values were obtained by chi-squared tests.

The mean number of natural teeth and POPs according to gender and age group are presented in Fig 1. In males, the mean number of natural teeth was 21.0 ± 0.29 in participants in their 60s, 17.1 ± 0.39 in their 70s, and 13.4 ± 0.76 in their 80s or older. In females, the mean number of natural teeth was 22.6 ± 0.21 in those in their 60s, 18.1 ± 0.33 in their 70s, and 11.7 ± 0.70 in their 80s or older. The mean number of POPs in males was 6.3 ± 0.15 in those in their 60s, 4.3 ± 0.19 in their 70s, and 2.7 ± 0.32 in their 80s or older. In females, the mean number of POPs was 7.0 ± 0.14 in their 60s, 4.5 ± 0.16 in their 70s, and 2.0 ± 0.22 in their 80s or older. The mean number of natural teeth and POPs decreased significantly as age increased in both males and females (p < 0.001).

**Fig 1:** Decrease of the mean number of natural teeth and POPs with age. The number of (A) natural teeth and (B) POPs significantly decreased with age in both males and females (*P* < 0.001). POPs, pairs of opposing posterior teeth.

The proportion of those with low handgrip strength according to the number of POPs and the presence of a hopeless tooth are presented in Fig 2. With the same number of POPs, the presence of a hopeless tooth increased the proportion of those with low handgrip strength in both males and females. In males, when the POPs score was 12, the low handgrip strength ratio was 4.5% without hopeless teeth, but increased to 20.3% in the presence of a hopeless tooth. In those with 8–11 POPs, the low handgrip strength ratio was 7.7% without hopeless teeth, and 14.2% in the presence of a hopeless tooth. In those with 0–7 POPs, the low handgrip strength ratio was 11.3% without hopeless teeth, and 16.2% in the presence of a hopeless tooth (*P* < 0.001). In females as well, when the POPs score was 12, 8–11, and 0–7, without hopeless teeth, the low handgrip strength ratio was 16.2, 16.2, and 29.1, respectively, but in the presence of a hopeless tooth, it increased to 25.6, 35.4, and 34.0 (*P* < 0.001).

The article "Hopeless tooth and less posterior occlusion is related to a greater risk of low handgrip strength: A population-based cross-sectional study" was published in 2021. Journal: PLoS One.

**Fig 2:** Increased proportion of individuals with low handgrip strength in the presence of a hopeless tooth. Within a similar posterior occlusion, the presence of a hopeless tooth increased the proportion of those with low handgrip strength in both (A) males and (B) females.

Table 2 presents the results of logistic regression analysis according to the posterior occlusion and the presence of hopeless teeth. In males, even when the number of POPs was 12, if they had a hopeless tooth, the odds ratio (OR) was high in crude model, model 1, and model 2, respectively, at 5.38, 4.61, and 3.39, although the association with low handgrip strength disappeared in model 2. With 8–11 POPs, the association in crude model was higher when they had a hopeless tooth (OR = 3.48, 95% CI = 1.39–8.69) than when they had no hopeless teeth (OR = 1.75, 95% CI = 0.95–3.21). In the absence of hopeless teeth, the association disappeared in model 1, but in the presence of a hopeless tooth, the association persisted until model 2 (OR = 2.82, 95% CI = 1.06–7.52). With 0–7 POPs, the association with low handgrip strength persisted until model 2 regardless of whether or not a hopeless tooth was present. In this group as well, the odds ratio increased in the presence of a hopeless tooth (OR = 2.78, 95% CI = 1.42–5.47) compared to the absence of hopeless teeth (OR = 1.91, 95% CI = 1.02–3.59) in model 2. In the final model, it was found that when the POPs score was 8–11 and they had a hopeless tooth, the association with low handgrip strength was higher (OR = 2.82, 95% CI = 1.06–7.52) than when the number of POPs was 0–7 and they had no hopeless teeth (OR = 1.91, 95% CI = 1.02–3.59).

**Table 2:** Odds ratios (ORs) and 95% confidence intervals (CIs) for low handgrip strength according to POPs and the presence of hopeless tooth.

Posterior occlusion	Hopeless tooth	Male			Female		
		Crude model	Model 1	Model 2	Crude model	Model 1	Model 2
Complete (POPs 12)	-	1.00	1.00	1.00	1.00	1.00	1.00
	+	5.38 (1.12–25.73)	4.61 (1.05–20.11)	3.39 (0.84–13.67)	1.76 (0.54–5.80)	1.39 (0.52–3.74)	1.43 (0.48–4.27)
Good (POPs 8–11)	-	1.75 (0.95–3.21)	1.81 (0.98–3.35)	1.59 (0.84–3.02)	0.99 (0.67–1.46)	0.87 (0.58–1.31)	0.91 (0.60–1.37)
	+	3.48 (1.39–8.69)	2.95 (1.13–7.66)	2.82 (1.06–7.52)	2.83 (1.36–5.89)	1.74 (0.81–3.73)	1.78 (0.82–3.86)
Poor (POPs 0–7)	-	2.68 (1.57–4.62)	2.42 (1.39–4.21)	1.91 (1.02–3.59)	2.11 (1.53–2.91)	1.20 (0.86–1.67)	1.09 (0.76–1.55)
	+	4.07 (2.18–7.60)	3.45 (1.82–6.57)	2.78 (1.42–5.47)	2.66 (1.66–4.26)	1.41 (0.86–2.32)	1.27 (0.76–2.13)

Values are presented as odds ratio (95% confidence interval).

-: No hopeless teeth.

+: Presence of a hopeless tooth.

The article "Hopeless tooth and less posterior occlusion is related to a greater risk of low handgrip strength: A population-based cross-sectional study" was published in 2021. Journal: PLoS One.

Model 1: Crude model additionally adjusted for age, household income, and education level.

Model 2: Model 1 additionally adjusted for fasting blood glucose, BMI, hs-CRP, blood pressure, sedentary time, muscular exercise, drinking, smoking, and denture status.

Abbreviations: BMI, body mass index; CI, confidence interval; hs-CRP, high-sensitivity C-reactive protein; OR, odds ratio; POPs, pairs of opposing posterior teeth.

In females as well, the association with low handgrip strength was higher in the presence of a hopeless tooth than no hopeless teeth. When the POPs was 8–11 and there was a hopeless tooth, it was associated with low handgrip strength (OR = 2.83, 95% CI = 1.36–5.89). For 0–7 POPs, the association remained regardless of the presence or absence of a hopeless tooth, and the odds ratio increased in the presence of a hopeless tooth (OR = 2.66, 95% CI = 1.66–4.26) compared to the absence of hopeless teeth (OR = 2.11, 95% CI = 1.53–2.91) in crude model. In females, the association disappeared in model 1, unlike in males.

Table 3 presents the association with low handgrip strength according to other characteristics of subjects from the multivariable adjusted logistic regression analysis. As the age increased, the OR significantly increased in both males and females. When Hs-CRP was higher than normal, the OR significantly increased only in females. As for sedentary time, when it was 7.4 or more hours per day in males and 4.7–9.9 hours per day in females, the risk of low grip strength significantly increased.

**Table 3:** Multivariable adjusted logistic regression analysis for evaluating the association with low handgrip strength according to other characteristics of subjects.

Variables		Male		Female	
		Model 1	Model 2	Model 1	Model 2
Age (years old)	60–69	1.00	1.00	1.00	1.00
	70–69	3.53 (2.38–5.24)	3.01 (1.99–4.55)	2.88 (2.24–3.68)	2.61 (2.01–3.40)
	≥80	17.62 (10.92–28.42)	11.86 (7.06–11.89)	8.18 (5.60–11.95)	6.66 (4.45–9.96)
Household income	Low	1.00	1.00	1.00	1.00
	Middle-low	1.02 (0.65–1.58)	1.06 (0.67–1.68)	0.95 (0.69–1.30)	0.96 (0.70–1.32)
	Middle-high	0.85 (0.54–1.36)	0.88 (0.55–1.42)	0.91 (0.66–1.25)	0.91 (0.66–1.26)
	High	0.85 (0.51–1.42)	0.95 (0.56–1.62)	0.71 (0.51–0.98)	0.72 (0.52–0.99)
Education level	Elementary school	1.00	1.00	1.00	1.00
	Middle school	0.48 (0.31–0.77)	0.47 (0.29–0.75)	0.77 (0.55–1.07)	0.83 (0.59–1.16)
	High school	0.45 (0.29–0.71)	0.48 (0.31–0.76)	0.45 (0.30–0.67)	0.44 (0.29–0.66)
	College or higher	0.38 (0.20–0.72)	0.36 (0.19–0.70)	0.81 (0.49–1.33)	0.79 (0.47–1.30)
Fasting blood glucose	Normal		1.00		1.00
	Pre-diabetes		0.88 (0.61–1.27)		1.08 (0.84–1.87)
	Diabetes		1.46 (0.91–2.36)		1.11 (0.79–1.57)
Body mass index (kg/m^2^)	<23		1.00		1.00
	23–25		0.65 (0.43–0.97)		0.61 (0.45–0.82)
	≥25		0.34 (0.21–0.54)		0.64 (0.49–0.83)
High-sensitivity C-reactive protein	Normal		1.00		1.00
	High		1.06 (0.74–1.52)		1.36 (1.07–1.73)
Blood pressure	Normal		1.00		1.00
	Pre-hypertension		0.58 (0.33–1.01)		1.28 (0.88–1.87)
	Hypertension		0.94 (0.60–1.47)		1.28 (0.92–1.78)
Sedentary time (hours/day)	<4.7		1.00		1.00
	4.7–7.4		1.42 (0.84–2.41)		1.45 (1.02–2.08)
	7.4–9.9		1.91 (1.10–3.29)		1.64 (1.09–2.46)
	≥9.9		2.00 (1.21–3.31)		1.32 (0.92–1.89)
Muscular exercise (days/week)	≤2		1.00		1.00
	3–4		1.50 (0.64–3.51)		1.17 (0.45–3.01)
	≥5		1.53 (0.89–2.62)		1.53 (0.79–2.96)
Drinking (glasses at a sitting)	None		1.00		1.00
	1–4		0.64 (0.43–0.93)		0.74 (0.58–0.94)
	5–9		0.46 (0.27–0.78)		0.37 (0.13–1.05)
	≥10		0.74 (0.25–2.21)		0.22 (0.03–1.74)
Smoking	Non-smoker		1.00		1.00
	Former smoker		0.74 (0.48–1.14)		1.23 (0.59–2.55)
	Current smoker		0.82 (0.46–1.14)		1.20 (0.60–2.41)
Denture status	No		1.00		1.00
	Yes		1.23 (0.81–1.88)		1.14 (0.85–1.54)

Values are presented as odds ratio (95% confidence interval).

The article "Hopeless tooth and less posterior occlusion is related to a greater risk of low handgrip strength: A population-based cross-sectional study" was published in 2021. Journal: PLoS One.

Abbreviations: BMI, body mass index; CI, confidence interval; hs-CRP, high-sensitivity C-reactive protein; OR, odds ratio; POPs, pairs of opposing posterior teeth.

## Discussion

In this study, we showed that the presence of hopeless teeth and less posterior occlusion were associated with low handgrip strength in this study. And, since the posterior occlusion is directly related to the masticatory function, the posterior occlusion was subdivided and analyzed to evaluate the effect of the hopeless tooth within a similar posterior occlusion.

Our results showed that the number of POPs decreased with age statistically significantly. Also, with a given number of POPs, the risk of low handgrip strength was significantly increased when a hopeless tooth was present in the dentition. In men, specifically, this association persisted even after adjustment for all confounding variables. When the number of POPs was 0–7, that is, poor condition for chewing, the risk of low handgrip strength was significantly higher regardless of the possession of a hopeless tooth, and, also with low POPs, the presence of a hopeless tooth increased the risk from 1.91 times to 2.78 times compared to the absence of it. It is interesting to note that men have a 2.82-fold higher risk of low handgrip strength when hopeless teeth are included in the dentition, even in cases in which they have enough posterior teeth for mastication (POPs ≥8). Moreover, this is even higher risk (OR = 2.82) than those with a dentition that lacks posterior teeth to the extent of poor masticatory function (POPs 0–7) without hopeless teeth (OR = 1.91). This implies that the hopeless teeth have a significant adverse effect on handgrip strength even before they are extracted.

The article "Hopeless tooth and less posterior occlusion is related to a greater risk of low handgrip strength: A population-based cross-sectional study" was published in 2021. Journal: PLoS One.

This association can be explained by several plausible mechanisms, the first being the mastication and nutritional component. Individuals with subjective chewing difficulty are prone to choose soft foods rather than hard foods such as meat, fruits, and vegetables, leading to lower intake of protein, vitamins, and minerals, and higher intake of carbohydrates, saturated fat, trans fat, and cholesterol [26–28]. Sufficient protein intake has been emphasized for the prevention and management of sarcopenia [29,30], and a review also described the importance of vitamin D, antioxidants, and unsaturated fatty acids [31]. Second is the neural mechanism. An association between orofacial and limb motoneuronal control has been demonstrated, and some studies have found that proprioception in the orofacial region may affect muscle strength [32]. Third, inflammatory mediators caused by hopeless teeth can continuously affect the muscles. Muscle degradation is promoted by pro-inflammatory cytokines such as IL-6 and TNF-alpha [33], which are well-established cytokines found in inflamed periodontal or pulp tissue [34–36]. In addition, elevated plasma oxidative status in periodontitis [37,38] may cause dysfunctional proteins to accumulate in skeletal muscle due to an increase in oxidative protein, leading to a decrease in muscle strength [39].

The association was found to be less significant in females, and there have been other studies showing similar tendencies [9,10,14]. A possible explanation is that both oral health and sarcopenia are greatly influenced by socioeconomic factors [9], and women are socially more vulnerable in terms of income and education [14]. In our results, the significance disappeared in a model adjusted for age, household income, and education level. An additional explanation for the gender difference is that women are more likely to have hopeless teeth extracted early to undergo prosthetic treatment for aesthetic reasons, whereas men are more likely to retain hopeless teeth for a long time, which can have a detrimental effect on muscle mass and strength [9]. Our results also showed that the mean number of hopeless teeth and the proportion of individuals with hopeless teeth were higher in men than in women.

The article "Hopeless tooth and less posterior occlusion is related to a greater risk of low handgrip strength: A population-based cross-sectional study" was published in 2021. Journal: PLoS One.

Another notable finding is that the average number of natural teeth and POPs are too small. For successful oral aging, the common goal of the World Health Organization and the Federation Dentaire Internationale is to maintain 20 or more natural teeth [1,20]. Ueno et al. reported that having 20 or more natural teeth and more than 7.6 natural FTU is important for masticatory ability [19]. However, the oral health of the elderly in Korea is in a state far below these goals. It follows that efforts to preserve natural teeth are needed at all levels, from the individual to dental care to health policy.

This study has several limitations. First, it was not possible to evaluate artificial tooth occlusion, because the KNHANES data did not include information on the restoration of individual teeth after extraction. Second, the results may vary depending on the position of hopeless teeth, but the samples with hopeless teeth in the anterior region were insufficient to be analyzed. Third, since it is a cross-sectional study, a causal relationship cannot be identified. Fourth, discomfort, such as pain or mobility, may be more relevant to the decrease in handgrip strength, but the symptoms of individual teeth were not examined in the KNHANES. Overall, further studies with a prospective design that examine the effect of symptoms of teeth, including functional teeth will be required to address aforementioned limitations.

Nevertheless, this study has several strong points. First, previous studies on the relationship with handgrip strength did not evaluate the condition of teeth, but in this study, we confirmed that it was insufficient to evaluate using only the number of remaining teeth, and it was important to consider the condition of the teeth. Even with a sufficient number of posterior teeth, the presence of hopeless teeth significantly increased the risk of low handgrip strength. Second, the posterior occlusion was evaluated with POPs, which better reflect the masticatory function, compared to evaluating only with the number of residual teeth. Moreover, unlike most previous studies intended to include only well-functioning teeth related to mastication, this study focused on severely compromised teeth and raised awareness of the role of hopeless teeth as well as fewer POPs in low handgrip strength. Overall, our findings collectively indicate the importance of preserving the posterior teeth in a healthy condition through thorough personal oral hygiene care and regular dental management to maintain physical functioning.
